The article "The Effect and Mechanism of Burnet Gels on Steroid-Dependent Dermatitis in Guinea Pig Model" was retracted in 2023. Reasons: signs of a paper mill; compromised peer review; unreliable results or conclusions.

# The Effect and Mechanism of Burnet Gels on Steroid-Dependent Dermatitis in Guinea Pig Model

**DOI:** 10.1155/2022/5866824

**Published:** 2022-09-13

**Authors:** Wenli Ma, Xiaojuan Ma, Xiaofan Li, Xuebin Xi, Chunyang Mao, Lixin Wang

**Affiliations:** ^1^Ningxia Medical University, Yinchuan, Ningxia 750004, China; ^2^Ningxia Minority Medicine Modernization Key Laboratory of Ministry of Education, Yinchuan, Ningxia 750004, China

## Abstract

**Objective:**

This study was designed to establish quality standards of Burnet gels and investigate the effects and mechanism of Burnet gels on steroid-dependent dermatitis (HDD) in guinea pigs.

**Methods:**

HPLC was used to determine the content of gallic acid, Gentiopicrin, and paeonol. A total of 48 male guinea pigs were recruited and randomly divided into control group, model group, tacrolimus ointment group, and Burnet gel group (Low, medium, and high concentration). The HDD guinea pig model was established by the 0.5% clobetasol propionate tincture. After HDD model establishment, control group and model group smeared normal saline and the rest of the group with corresponding drugs for three weeks. The contents of IFN-*γ*, IL-4, and IgE in the guinea pig serum were detected by the ELISA; the protein expression levels of FLG, LOR, and Caspase-14 in the epidermis of guinea pigs were detected by the immunohistochemical and Western blotting method.

**Results:**

The content of gallic acid, Gentiopicrin, and paeonol was 0.30 mg/g, 1.06 mg/g, and 0.56 mg/g. Compared with the normal group, the IFN-*γ*, IL-4, and IgE of guinea pig serum in the model group were significantly increased; the FLG, LOR, and Caspase-14 of guinea pig epidermis in the model group were significantly decreased; compared with the model group, the IFN-*γ*, IL-4, and IgE of guinea pig serum in the tacrolimus ointment group and Burnet gel group were significantly decreased; the FLG, LOR, and Caspase-14 of guinea pig epidermis in the tacrolimus ointment group and Burnet gel group were significantly increased.

**Conclusion:**

Burnet gels can improve guinea pig HDD model, and the mechanism may be related to inhibiting skin inflammation and promoting the formation of epidermal skin barrier.

## 1. Introduction

Glucocorticoids are widely used in the treatment of various skin diseases due to their multiple functions such as inhibiting proliferation, inhibiting immunity, anti-inflammatory, and whitening [1, 2]. After long-term use, drug withdrawal is likely to induce withdrawal reactions, which manifest as local skin erythema, acne, desquamation, and dryness at the skin lesions, accompanied by local tingling, burning, itching, and other rosacea-like changes. It can be relieved, making patients physically and psychologically dependent [3, 4]. According to reports, this hormone-dependent dermatitis (HDD) induced by long-term use of hormones often occurs 5-7 days after the withdrawal of hormone preparations, which seriously affects the physical and mental health of patients [5]. The skin barrier is a dense structure formed by the cross-linking of the protein envelope expressed by keratinocytes and the intercellular lipid envelope. It is distributed in the outermost layer of the skin epidermis. It plays an important role in the homeostasis of the body's internal environment and in resisting the invasion of foreign substances [6].

The article "The Effect and Mechanism of Burnet Gels on Steroid-Dependent Dermatitis in Guinea Pig Model" was retracted in 2023. Reasons: signs of a paper mill; compromised peer review; unreliable results or conclusions.

Loricrin (LOR) is the most important protein in the skin barrier, and its content accounts for 80% of the total protein in the stratum corneum [7]. Another key protein, filaggrin (FLG), is processed by cysteine protease-14 (Caspase-14), cut and catabolize into free amino acids, provide skin with natural moisturizing factors, and maintain skin moisture [8]. HDD is characterized by disruption of skin barrier-associated proteins, and with the disruption of the skin barrier, a keratinocyte-derived inflammatory cascade is initiated, and T helper cells and eosinophils are increased [9, 10].

Burnet gel is a prescription for clinical experience. It is composed of Burnet, Gentian, Sophora Radix, Cortex Moutan, Licorice, Licorice, and other traditional Chinese medicines. The effect of facial dermatitis is obvious [11, 12], but the quality standard and related pharmacodynamics research for this gel is still lacking. In this study, on the basis of establishing the quality standard of Burnet gel, the HDD guinea pig model was intervened, and its mechanism of action was discussed from the perspective of regulating immunity and skin barrier repair mechanism and provided theoretical support for clinical medication.

## 2. Methods

### 2.1. Animals

48 healthy 2-month-old female albino guinea pigs, weighing 330 ± 20 g, were purchased from the Experimental Animal Center of Ningxia Medical University (license number: SYXK (Ning) 2020-0001). The experimental study has been reviewed by the Animal Ethics Committee of Ningxia Medical University (approval code: IACUC-NYLAC-2021-053).

### 2.2. Drugs

Burnet (batch: 20210201), gentian (batch: 20210201), Sophora flavescens (batch: 20210201), Cortex Moutan (batch: 20210201), purple herb (batch: 20210201), and the licorice herbs (batch number: 20210201) were purchased from Ningxia Mingde Chinese Medicine Decoction Pieces Co., Ltd.; standard products, gallic acid (production batch number: 110831-201906), gentiopicroside (production batch number: 110770-201918), and paeonol (production batch number: 110770-201918) (batch numbers: 110708-201908), were purchased from China National Institute for Food and Drug Control; Burnet gel (made by the Key Laboratory of Modernization of Minority Medicine, Ningxia Medical University, 20210915, 20211002, 20211008); clobetasol propionate (China Food and Drug Administration) (Inspection Institute, batch number: 100302-201804); 0.03% tacrolimus ointment (Zhejiang Wansheng Pharmaceutical Co., Ltd.).

The article "The Effect and Mechanism of Burnet Gels on Steroid-Dependent Dermatitis in Guinea Pig Model" was retracted in 2023. Reasons: signs of a paper mill; compromised peer review; unreliable results or conclusions.

### 2.3. Reagents

Reagents are as follows: purified water (Wahaha Group); acetonitrile (chromatographic grade, Fisher Scientific); methanol (chromatographic grade, Yuwang Industrial Co., Ltd.); IL-4 (JL21520), IFN-*γ* (JL11665), IgE (JL11287) ELISA kits (Shanghai Jianglai Biotechnology Co., Ltd.); FLG (Affinity, USA, DF13653); LOR (Thermo Fisher Scientific, USA); Caspase-14 (Novus, USA); 0.25% trypsin protein digestion solution (Beijing Soleibao Technology Co., Ltd., T1350); goat anti-rabbit secondary antibody, goat anti-mouse secondary antibody, DAB color reagent, ECL luminescence kit (Beijing Zhongshan Jinqiao Biotechnology Co., Ltd., ZB2301, ZB2305, ZLI-9018, SC-2048); hematoxylin staining solution (Zhuhai Besuo Biotechnology Co., Ltd., BA-4041). The second antibodies goat anti-rabbit IgG (H+L) HRP (FMS-Rb01, Fcmacs) and goat anti-mouse IgG (H+L) HRP (S0002, Affinity) were in 5000 diluted concentrations.

### 2.4. Experimental Instruments

The experimental instruments are as follows: AL204 electronic balance (*d* = 0.1 mg, Shanghai METTLER TOLEDO Instrument Co., Ltd.); LC-2030C high-performance liquid chromatograph (Shimadzu Corporation of Japan); ultratrace UV-Vis spectrophotometer DS-11 (Danoer, USA); BP310P weighing balance (Sartorius, Germany); Centrifuge5417R low-temperature high-speed centrifuge (Eppendorf, Germany); KX-ZOON400 Yaoguang infrared scientific research system (Shandong Yaoguang Medical Technology Co., Ltd.).

## 3. Methods and Results

### 3.1. Establishment of Quality Standards for Burnetia Chinensis Gel (Determination of Content)

#### 3.1.1. Preparation of Solution

*(1) Mixed Reference Solution.* Add methanol to make single reference substance mother liquor with mass concentrations of 0.7128 mg/mL, 1.4107 mg/mL, and 1.3976 mg/mL, respectively. Take appropriate amount of methanol to make gallic acid, gentiopicroside, and paeonol with mass fractions of mixed reference solution of 0.0394 mg/mL, 0.1576 mg/mL, and 0.0788 mg/mL.

*(2) Test Solution.* Precisely weigh 1 g of Burnet gel under item “2.2” in a 25 mL volumetric flask, add methanol to 25 mL, extract ultrasonically until the solution is turbid, add methanol to the volume, shake well, and draw 1.8 mL. This solution was placed in a 2 mL centrifuge tube, centrifuged, and the supernatant part of the tube was collected as the test solution.

*(3) Negative Solution.* Prepare gallic acid, gentiopicroside, and paeonol negative solution according to the preparation method of Burnet gel solution under “3.1.1(2).”

The article "The Effect and Mechanism of Burnet Gels on Steroid-Dependent Dermatitis in Guinea Pig Model" was retracted in 2023. Reasons: signs of a paper mill; compromised peer review; unreliable results or conclusions.

#### 3.1.2. Chromatographic Conditions

Chromatographic column (model: Agilent TC-C18, size: 4.6 mm × 250 mm, 5 *μ*m), mobile phase conditions: acetonitrile (A)-0.1% phosphoric acid aqueous solution (B), gradient elution, detector wavelength: 254 nm, flow rate: 1.0 mL/min, column oven temperature 30°C, and sample injection volume 10 *μ*L. The specific gradient elution procedure is shown in Table 1.

#### 3.1.3. Methodological Evaluation

*(1) Specificity Test.* According to the chromatographic conditions under “3.1.2,” accurately draw 10 *μ*L of the 5 solutions under “3.1.1” and inject samples for measurement, and record the chromatograms in sequence. Results: the chromatographic peaks of gallic acid, gentiopicroside, paeonol, and their adjacent peaks all achieved baseline separation; the resolution was all ≥1.5, the negative control had no interference, and the number of theoretical plates was ≥3000 (with gallic acid, peak meter) (see Figure 1).

### 3.2. Linear Relationship Investigation

Precisely add 1.0 mL each of the mother solutions of the three single reference substances under “3.1.1(1)” into a 5 mL volumetric flask, dilute to the mark with methanol, and shake well. Precisely draw 1.0 mL, dilute 5, 10, 15, 20, and 25 times with methanol solution to prepare 5 groups of mixed reference solutions with a linear relationship, inject samples under the chromatographic conditions in “3.1.2,” and measure and record the chromatogram picture. Taking the injection concentration (C) of each group as the abscissa and the ordinate as the peak area (Y), the linear regression analysis was performed to obtain the linear regression equations of the three components; the signal-to-noise ratio (S/N) was 3 : 1, respectively. With 10 : 1 as the detection benchmark, the detection limit and quantification limit of each component to be tested were calculated, and the results are shown in Table 2.

#### 3.2.1. Precision Test

According to the above chromatographic conditions, accurately draw 10 *μ*L of the test solution into the sample, repeat 6 times in a row, and calculate the RSD value by measuring the peak area of each component. Results: the RSDs of the peak areas of gallic acid, gentiopicroside, and paeonol were 1.65%, 1.81%, and 0.39%, respectively, indicating that the precision of the instrument was good.

*(1) Repeatability Test.* Prepare 6 samples of Burnet elm gel in parallel, prepare 6 solutions in parallel according to the same method in “3.1.1(2),” inject samples under the above chromatographic conditions, and measure and record the chromatogram. Results: the average contents of gallic acid, gentiopicroside, and paeonol were measured as 0.30 mg/g, 1.06 mg/g, and 0.56 mg/g, and the RSD values of the contents were 1.84%, 1.69%, and 1.55%, respectively.

*(2) Stability Test.* Take the same batch of the test solution, place it at room temperature, and inject the sample under the above chromatographic conditions after 0, 2, 12, 16, 18, and 24 hours, respectively, and measure and record the chromatogram. Results: the RSD values of the peak areas of gallic acid, gentiopicroside, and paeonol were 1.43%, 1.51%, and 0.60%, indicating that the sample was stable and reliable within 24 hours at room temperature.

*(3) Sample Addition Recovery Test.* 6 parts of 0.50 g Burnet gel are accurately weighed and placed in 25 mL volumetric flasks, and a separately prepared mixed reference solution (containing 0.1508 mg/mL gallic acid, gentiopicroside 0.5012 mg/mL, and paeonol 0.2801 mg/mL) 1.0 mL, according to the same method in “3.1.1(2)” to prepare 6 solutions in turn, inject samples under the above chromatographic conditions, and measure and record the chromatogram. The recovery rates of the above three main components were calculated, and the results are shown in Table 3.

The article "The Effect and Mechanism of Burnet Gels on Steroid-Dependent Dermatitis in Guinea Pig Model" was retracted in 2023. Reasons: signs of a paper mill; compromised peer review; unreliable results or conclusions.

### 3.3. Pharmacodynamics Study of Burnet Gel

#### 3.3.1. Method

*(1) Preparation of Burnet Gel with Different Concentration Gradients.* The proportion of extract was 2.5%, the middle-dose group of Burnet gel; the proportion of extract was 5%, the high-dose group of Burnet gel; the proportion of extract was 10%.

*(2) Establishment of HDD Guinea Pig Model.* 48 guinea pigs were selected from the left and right sides of the back to cut their hair in a 5 × 5 cm area, and the remaining hair was removed with depilatory cream. 8 guinea pigs were randomly selected as blank group, 75% alcohol was applied on the right side, 0.9% normal saline was applied on the left side, and the remaining 40 guinea pigs were applied with 0.05% clobetasol propionate tincture on the right side and 75% alcohol on the left side, 2 times a day. Second rate: the model was successfully replicated after 7 weeks [13].

*(3) Grouping and Administration.* The above 40 HDD model guinea pigs were randomly divided into 5 groups, namely, model group, positive control group, Burnet gel low-dose group, Burnet gel medium-dose group, and Burnet gel high-dose group. The right skin of the blank group and model group was smeared with 0.9% normal saline, the right skin of the gel treatment group was smeared with the corresponding gradient gel preparation, and the right skin of the positive control group was smeared with 0.03% tacrolimus ointment, twice a day for 3 consecutive weeks.

*(4) Detection of Sebum Tester, Dermoscopy, and Infrared Imaging System.* Using a sebum tester and dermoscopy, the bilateral skin of the above 6 groups of guinea pigs were tested before and after treatment, and the skin moisture and oil were repeatedly tested. The average value was taken as the skin moisture and oil content values; skin tissue images were collected by dermoscopy; bilateral skin temperature was measured by infrared imaging system.

*(5) Sample Collection.* The sample was collected 12 hours after the last administration; after intraperitoneal anesthesia with 3% sodium pentobarbital, blood was taken from the apex and centrifuged at 3500 r/min for 15 min, and the supernatant was taken and packed in cryovials and stored in -80°C refrigerator. The intact skin of the bilateral depilation area of guinea pigs was taken, part of which was fixed in 4% paraformaldehyde solution, and the remaining part was aliquoted in cryopreservation tubes and stored in a -80°C refrigerator.

*(6) Detection of Serum Inflammatory Factors.* Take the supernatant from “3.3.1(5),” and detect the levels of serum IL-4, IFN-*γ*, and IgE according to the instructions of the ELISA kit.

*(7) Pathological Detection of Skin Tissue.* The tissue after fixation with 4% paraformaldehyde solution in “3.3.1(5)” was routinely dehydrated, embedded in paraffin, sectioned (with a thickness of 5um), stained with HE, and then, mounted. The histomorphological changes were observed under a light microscope (×200).

*(8) Immunohistochemical Detection of FLG, LOR, and Caspase-14 Protein Expression in Skin Tissue.* Deparaffinize the sections to water, repair by antigen high pressure, incubate, block with serum, drop primary antibodies diluted with PBS, and place in a wet box. Incubate overnight at 4°C, wash 3 times with PBS, 5 min/time, add HRP-labeled secondary antibody dropwise, incubate at room temperature for 30 min, wash 3 times in the same way, add newly prepared DAB chromogenic solution to develop color, counterstain nuclei with hematoxylin, dehydrated, mounted, and observed under a microscope (×400), the nuclei were blue, and the positive expression was brown.

*(9) Western Blotting Method to Detect the Expression of FLG, LOR, and Caspase-14 in Skin Tissue.* Put the skin tissue in 0.25% trypsin protein digestion solution and soak it for 16 h at 4°C, gently peel off the epidermis, weigh 50 mg, and cut it into pieces, ground in liquid nitrogen to a fine powder, aliquoted into centrifuge tubes, added 500 ul of RIPA lysis solution, mixed well, placed at 4°C overnight, and centrifuged at 12000 rpm for 10 min at 4°C, and the supernatant was taken. The protein concentration was determined by ultratrace UV-Vis spectrophotometer and denatured at 95°C for 10 min. After loading on SDS-PAGE gel, electrophoresis, and PVDF transfer membrane, blocking with 5% nonfat milk powder at room temperature for 2 h, and adding primary antibody diluted with PBS, overnight at 4°C, and washed with PBST solution 3 times, 10 min/time, the secondary antibody diluted with PBST was added for 90 min. After washing with the same method, the ECL method was used to develop the film, and the film was scanned. Image-J software was used to measure the gray value of the band.

*(10) Statistical Methods.* SPSS 23.0 software was used to analyze the data. All measurement data were in line with normal distribution and were expressed in the form of mean ± standard deviation (□*x* ± *s*), and the data comparison between multiple groups used one-way variance analysis; *P* < 0.05 indicates a statistically significant difference.

The article "The Effect and Mechanism of Burnet Gels on Steroid-Dependent Dermatitis in Guinea Pig Model" was retracted in 2023. Reasons: signs of a paper mill; compromised peer review; unreliable results or conclusions.

## 4. Results

### 4.1. Comparison of Skin Moisture, Oil Content, and Skin Temperature of Guinea Pigs in Each Group

Compared with the blank group, the skin moisture and oil content of the model group decreased significantly, and the skin temperature increased (*P* < 0.01); compared with the model group, the skin moisture and oil content of the Burnet gel medium- and high-dose groups and the tacrolimus group increased, and the skin temperature decreased (*P* < 0.05). Water and oil content gradually increased (Table 4).

### 4.2. Dermoscopic Characteristics of Guinea Pigs in Each Group

Compared with the blank group, the skin of guinea pigs in the model group showed telangiectasia, and the surface was covered with scattered scales; in the division group, scaling was regressed, and telangiectasia improved (Figure 2).

### 4.3. The Morphological Changes of the Guinea Pig Skin in Each Group

Compared with the blank group, the model group guinea pigs showed parakeratosis of the epidermis, hyperplasia of the epidermis, acanthosis, the epidermis descended in a club-like shape, and the superficial dermis was densely inflammatory cell infiltration; compared with the model group, the stratum corneum mesh basket thickening, epidermal hyperplasia, and inflammatory cell infiltration in the superficial dermis were improved in the medium- and high-dose groups of Burnet gel and the tacrolimus group (Figure 3).

### 4.4. Changes in the Levels of IL-4, IFN-*γ*, and IgE in the Serum of Guinea Pigs in Each Group

Compared with the blank group, the levels of IL-4, IFN-*γ*, and IgE in the serum of guinea pigs in the model group were all increased, and the difference was statistically significant (*P* < 0.01); compared with the model group, the levels of IL-4, IFN-*γ*, and IgE in the serum of guinea pigs in the high-dose Burnet gel group and the tacrolimus group were decreased, and the difference was statistically significant (*P* < 0.05), and with the increase of gel concentration, the levels of IL-4 and IgE in guinea pig serum gradually decreased (Table 5).

The article "The Effect and Mechanism of Burnet Gels on Steroid-Dependent Dermatitis in Guinea Pig Model" was retracted in 2023. Reasons: signs of a paper mill; compromised peer review; unreliable results or conclusions.

### 4.5. Protein Expression of FLG, LOR, and Caspase-14 in the Epidermal Tissue of Guinea Pigs in Each Group

Immunohistochemical results showed that FLG, LOR, and Caspase-14 were mainly expressed in the epidermal stratum corneum, granular layer, and around the hair follicles of the dermis (Figure 4). The results of Western blotting method (Figure 5) showed that compared with the blank group, the expression of FLG, LOR, and Caspase-14 in the epidermis of the model group was significantly downregulated (*P* < 0.01); the expression of FLG, LOR, and Caspase-14 was significantly upregulated in the dose group and tacrolimus group (*P* < 0.05).

## 5. Discussion

The pathogenesis of HDD is not fully understood, but it is mainly believed to be related to the breakdown of the skin barrier. Long-term topical application of corticosteroids inhibits normal epidermal differentiation and reduces the synthesis of structural components of epidermal terminal differentiation, such as total protein and fibrillin, ultimately causing skin barrier function defects [10]. The results of this study showed that after 7 weeks of topical clobetasol propionate, the model was successfully established, the epidermal tissue-related proteins FLG, LOR, and Caspase-14 were downregulated, transdermal water loss (TEWL) increased, skin moisture, decreased oil content, manifested as dryness, desquamation, etc.

Acute-phase HDD skin is characterized by overexpression of the Th2 cytokines IL-4 and IgE. Studies have confirmed that in the early stage of stratum corneum skin barrier damage, unknown antigens or allergens activate IL-4 to convert Th0 cells into Th2 cells and migrate to the skin. Secrete more Th2 cytokines and other proinflammatory factors. In the late stage, a large amount of Th1 cytokines such as IFN-*γ* is induced, which also further promotes the inflammatory process and leads to late (chronic) skin damage. In the absence of strong inhibitory mechanisms, this inflammatory process may continue indefinitely [14, 15]. In this study, the local skin symptoms of HDD guinea pigs were aggravated after the hormone preparation was stopped, and the levels of serum IL-4, IgE, and IFN-*γ* were significantly higher than those of the blank control group.

The article "The Effect and Mechanism of Burnet Gels on Steroid-Dependent Dermatitis in Guinea Pig Model" was retracted in 2023. Reasons: signs of a paper mill; compromised peer review; unreliable results or conclusions.

The results of this study showed that the HDD guinea pig model showed hyperplasia of epidermis, parakeratosis in the stratum corneum, and decreased expression of epidermis-related proteins, which may be related to the formation of inflammatory cascades. IL-4 and IFN-*γ* can induce the apoptosis of HDD keratinocytes to increase and damage the skin barrier, reduce the expression of FLG, LOR, and Caspase-14 in the epidermis, continuously aggravate the degree of skin lesions, and prolong the duration of the skin lesions, causing the epidermis to increase thickness and parakeratosis [16–18].

Burnet gel is a compound preparation of traditional Chinese medicine. The types of traditional Chinese medicines contained in this preparation are relatively complex. Among them, paeonol, the main medicinal component of Cortex Moutan, is volatile. Accordingly, this study improved the extraction process of the main components in the prescription and used HPLC to investigate the content and stability of the main components of Burnet gel. The extraction methods used in traditional Chinese medicines are reliable and suitable for the extraction of the main active components of traditional Chinese medicines.

In present study, HPLC was used to determine the content of gallic acid, Gentiopicrin, and paeonol. HPLC is based on the principle of UV detection, which has the problems of low sensitivity and poor specificity. In LC/MS, mass spectrometer is used as the detection system, and specific selected ions are used as signal recording objects, so that the response to the target is higher, and the detection limit is lower. The detection specificity of the target is stronger. The use of LC-MS can not only avoid complicated, tedious, and time-consuming separation and purification work but also can separate and identify trace amounts of drug metabolites that were difficult to identify in the past, which can be quickly and easily applied to research. The screening of fragment ions by mass spectrometer enables a part of substances with similar polarities to be easily distinguished, so that analysts can use the same chromatographic conditions when separating substances with similar polarities, and in the case of poor separation, the analysis of samples that cannot be eliminated in the high performance liquid chromatography greatly improves the analysis efficiency. At the same time, with the continuous improvement of the instrument, the instrument has achieved a high degree of automation, which greatly reduces the workload of the analyst and improves the efficiency of the analysis. Therefore, we will employ LC-MS/MS to detect the content of gallic acid, Gentiopicrin, and paeonol.

The article "The Effect and Mechanism of Burnet Gels on Steroid-Dependent Dermatitis in Guinea Pig Model" was retracted in 2023. Reasons: signs of a paper mill; compromised peer review; unreliable results or conclusions.

In this study, Burnet gel was used to intervene in HDD guinea pig model, and it was found that it can significantly reduce serum IL-4 and IFN-*γ*. Epidermal thickness improves the state of epidermal hyperplasia. Compared with the blank control group, Burnet gel enhanced the expression of FLG, LOR, and Caspase-14 in epidermal tissue, promoted the formation of skin barrier, and reduced TEWL, and its mechanism of action may be related to the improvement of skin inflammation. In conclusion, Burnet gel can inhibit the occurrence of skin inflammation, reduce epidermal thickness, improve epidermal hyperplasia, restore the expression of damaged skin barrier-related proteins, and reduce TEWL. It can provide new ideas for the treatment of HDD.

## Figures and Tables

**Figure 1:** HPLC chromatograms of (a) testing sample, (b) mixed reference substances, (c) negative sample without Burnet and Moutan Cortex, (d) negative sample without Gentianae Radix et Rhizoma, and (e) negative sample without Moutan Cortex.(1. gallic acid; 2. Gentiopicrin; 3. paeonol).

**Figure 2:** Dermoscopy characteristics of guinea pigs in each group.

**Figure 3:** Morphological changes of guinea pig skin in each group (×200).

**Figure 4:** Immunohistochemical results of FLG, LOR, and Caspase-14 in guinea pig epidermis of each group (×400).

**Figure 5:** The expression of FLG, LOR, and Caspase-14 in guinea pig epidermis of each group detected by Western blot. Note: ^#^*P* < 0.05, ^##^*P* < 0.01, compared with the blank control group; ^∗^*P* < 0.05, ^∗∗^*P* < 0.01, compared with the model group.

**Table 1:** Gradient elution procedure.

Time (min)	A (%)	B (%)
0~4	7	93
4~8	7⟶11	93⟶89
8~15	11⟶12	89⟶88
15~20	12	88
20~25	12⟶13	88⟶87
25~45	13⟶65	87⟶35

**Table 2:** Regression equation and linear range.

Component	Regression equation	*r*	Linear range (ug/mL)	Detection limit (ug/mL)	The limit of quantitation (ug/mL)
Gallic acid	*y* = 19.535*x* − 1350.492	0.9996	5.70~28.51	0.3261	1.0871
Gentiopicroside	*y* = 11.913*x* − 1576.179	0.9996	11.29~56.43	0.8811	2.9371
Paeonol	*y* = 18.319*x* − 4387.861	0.9995	11.18~55.90	0.3668	1.2227

**Table 3:** Recovery rate results (*n* = 6).

Component	Weight/g	Sample size	Adding amount	Measured amount	Recovery rate	Mean	RSD
		mg			%		
Gallic acid	0.1484	0.1484	0.1508	0.2954	97.43	97.83	1.55
	0.1496	0.1496	0.1508	0.2917	94.22		
	0.1478	0.1478	0.1508	0.2917	95.41		
	0.1487	0.1487	0.1508	0.2957	97.46		
	0.1497	0.1497	0.1508	0.2960	97.03		
	0.1483	0.1483	0.1508	0.2905	94.33		

Gentiopicroside	0.5312	0.5312	0.5012	1.0257	98.66	97.83	1.83
	0.5353	0.5353	0.5012	1.0194	96.57		
	0.5290	0.5290	0.5012	1.0148	96.94		
	0.5323	0.5323	0.5012	1.0364	100.58		
	0.5358	0.5358	0.5012	1.0150	95.63		
	0.5306	0.5306	0.5012	1.0247	98.58		

Paeonol	0.2798	0.2798	0.2801	0.5445	94.47	96.09	1.44
	0.2820	0.2820	0.2801	0.5490	95.31		
	0.2787	0.2787	0.2801	0.5539	98.25		
	0.2804	0.2804	0.2801	0.5525	97.15		
	0.2823	0.2823	0.2801	0.5474	94.66		
	0.2795	0.2795	0.2801	0.5503	96.69		

The article "The Effect and Mechanism of Burnet Gels on Steroid-Dependent Dermatitis in Guinea Pig Model" was retracted in 2023. Reasons: signs of a paper mill; compromised peer review; unreliable results or conclusions.

**Table 4:** Comparison of water content, oil content, and skin temperature of guinea pigs in each group (*x* ± *s*, *n* = 8).

Groups	The proportion of drugs (%)	Moisture (%)	Oil (%)	Temperature (°C)
Blank control	—	29.78 ± 1.72	42.33 ± 3.85	33.80 ± 0.40
Model group	—	20.50 ± 1.87^##^	25.56 ± 5.02^##^	34.87 ± 0.39^##^
Gel low-dose group	2.5	26.88 ± 5.29^∗^	29.04 ± 2.33	34.36 ± 0.29^∗^
Gel mid-dose group	5	27.42 ± 4.17^∗∗^	32.67 ± 3.12^∗∗^	34.38 ± 0.21^∗^
Gel high-dose group	10	29.48 ± 1.79^∗∗^	38.86 ± 4.45^∗∗^	34.43 ± 0.23^∗^
Tacrolimus group	0.03	25.21 ± 4.28^∗^	38.63 ± 6.23^∗∗^	34.23 ± 0.44^∗^

Note: compared with the blank group, ^#^*P* < 0.05, ^##^*P* < 0.01; compared with the model group, ^∗^*P* < 0.05, ^∗∗^*P* < 0.01, the same below.

**Table 5:** Changes of IL-4, IFN-*γ*, and IgE levels in serum of guinea pigs in each group.

Groups	IL-4 (pg/mL)	IFN-*γ* (pg/mL)	IgE (*μ*g/mL)
Blank control	7.95 ± 0.49	8.25 ± 1.49	43.37 ± 6.28
Model group	10.54 ± 0.48^##^	14.37 ± 1.57^##^	60.29 ± 2.98^##^
Gel low-dose group	9.68 ± 1.49	12.69 ± 2.03	57.22 ± 4.86
Gel mid-dose group	8.98 ± 0.98^∗^	13.79 ± 1.23	55.65 ± 7.04
Gel high-dose group	8.84 ± 0.70^∗∗^	10.38 ± 1.04^∗∗^	52.59 ± 3.66^∗^
Tacrolimus group	7.84 ± 0.51^∗∗^	10.43 ± 2.07^∗^	41.71 ± 3.51^∗∗^

Note: ^#^*P* < 0.05, ^##^*P* < 0.01 compared with the blank control group; ^∗^*P* < 0.05, ^∗∗^*P* < 0.01 compared with the model group.

## Data Availability

All data, models, and code generated or used during the study appear in the submitted article.

## References

[1] Gabros S., Nessel T. A., Zito P. M. (2021). *Topical corticosteroids*.

[2] Jhaj R., Asati D. P., Chaudhary D., Sadasivam B. (2021). Topical steroid containing combinations: burden of adverse effects and why the recent regulatory action may not be enough. *Indian Journal of Pharmacology*.

[3] Lahiri K., Coondoo A. (2016). Topical steroid damaged/dependent face (TSDF): an entity of cutaneous pharmacodependence. *Indian Journal of Dermatology*.

[4] Sheary B. (2018). Steroid withdrawal effects following long-term topical corticosteroid use. *Dermatitis*.

[5] Rastogi M. K., Mohan R., Gahalaut P., Mishra N., Thapa M. (2019). Effect of topical steroid-dependent facial dermatitis on quality of life: a hospital-based cross-sectional study using DLQI. *Indian Journal of Dermatology*.

[6] Chambers E. S., Vukmanovic S. M. (2020). Skin barrier immunity and ageing. *Immunology*.

The article "The Effect and Mechanism of Burnet Gels on Steroid-Dependent Dermatitis in Guinea Pig Model" was retracted in 2023. Reasons: signs of a paper mill; compromised peer review; unreliable results or conclusions.

[7] Kim B. E., Leung D. Y. (2012). Epidermal barrier in atopic dermatitis. *Allergy, Asthma & Immunology Research*.

[8] Hoste E., Kemperman P., Devos M. (2011). Caspase-14 is required for filaggrin degradation to natural moisturizing factors in the skin. *The Journal of Investigative Dermatology*.

[9] Mandlik D. S., Mandlik S. K. (2021). Atopic dermatitis: new insight into the etiology, pathogenesis, diagnosis and novel treatment strategies. *Immunopharmacology and Immunotoxicology*.

[10] Lin T., Wei K., Wu C. (2015). Barrier abnormalities and keratinocyte-derived cytokine cascade after cessation of long-term topical glucocorticosteroid on hairless mouse skin. *Dermatologica Sinica*.

[11] Xiaocen Z. (2016). *Clinical observation on the treatment of facial dermatitis by oral administration of traditional Chinese medicine combined with external application of self-made Amaranth wet compress prescription*.

[12] Xiaolin Z. (2019). *Experimental study*.

[13] Weihua P., Hai W., Xiaogang L., Yuli L. (2005). Establishment of a guinea pig hormone-dependent dermatitis model and dynamic observation of skin changes. *China Aesthetic Medicine*.

[14] Chen L., Martinez O., Overbergh L., Mathieu C., Prabhakar B. S., Chan L. S. (2004). Early up-regulation of Th2 cytokines and late surge of Th1 cytokines in an atopic dermatitis model. *Clinical and Experimental Immunology*.

[15] Sung Y., Yuk H., Yang W., Kim S. H., Kim D. S. (2020). Siraitia grosvenorii residual extract attenuates atopic dermatitis by regulating immune dysfunction and skin barrier abnormality. *Nutrients*.

[16] Nakahara T., Mitoma C., Hashimoto-Hachiya A. (2015). Antioxidant Opuntia ficus-indica extract activates AHR-NRF2 signaling and upregulates filaggrin and loricrin expression in human keratinocytes. *Journal of Medicinal Food*.

[17] Sirobhushanam S., Parsa N., Reed T. J. (2020). Staphylococcus aureus colonization is increased on lupus skin lesions and is promoted by IFN-mediated barrier disruption. *The Journal of Investigative Dermatology*.

[18] Hong S., Lee B., Kim J. (2020). Solanum nigrum Linne improves DNCB-induced atopic dermatitis-like skin disease in BALB/c mice. *Molecular Medicine Reports*.

